The article "CAW: A Remote-Sensing Scene Classification Network Aided by Local Window Attention" was published in 2022. Journal: Comput Intell Neurosci.

# CAW: A Remote-Sensing Scene Classification Network Aided by Local Window Attention

**DOI:** 10.1155/2022/2661231

**Published:** 2022-10-11

**Authors:** Wei Wang, Xiaowei Wen, Xin Wang, Chen Tang, Jiwei Deng

**Affiliations:** School of Computer and Communication Engineering, Changsha University of Science and Technology, Changsha 410114, China

## Abstract

Remote-sensing image scene data contain a large number of scene images with different scales. Traditional scene classification algorithms based on convolutional neural networks are difficult to extract complex spatial distribution and texture information in images, resulting in poor classification results. In response to the above problems, we introduce the vision transformer network structure with strong global modeling ability into the remote-sensing image scene classification task. In this paper, the parallel network structure of the local-window self-attention mechanism and the equivalent large convolution kernel is used to realize the spatial-channel modeling of the network so that the network has better local and global feature extraction performance. Experiments on the RSSCN7 dataset and the WHU-RS19 dataset show that the proposed network can improve the accuracy of scene classification. At the same time, the effectiveness of the network structure in remote-sensing image classification tasks is verified through ablation experiments, confusion matrix, and heat map results comparison.

## 1. Introduction

With the development of satellite remote-sensing technology and unmanned aerial vehicle technology, the intersection of remote sensing and computer vision provides a new research area for remote-sensing image processing. Compared to terrestrial imagery, remote-sensing imagery provides a different perspective to describe the Earth's surface and facilitate a range of Earth observation missions [1]. Remote-sensing image scene classification is the fundamental work for understanding remote-sensing imagery and plays an important role in remote-sensing imagery applications such as Land Use/Land Cover (LULC) classification [2–4] and urban planning [5].

Remote-sensing image scene classification refers to the classification of different remote-sensing images in a dataset according to certain classification features, so the key to scene classification lies in the extraction of image features. The following are three types of methods for image feature extraction: First, the feature descriptors are directly extracted from the image, such as color histogram, scale-invariant feature transform SIFT [6], directional gradient histogram HOG [7], and local binary pattern LBP; the second is to continue feature extraction based on some underlying features extracted from image blocks, such as the bag-of-words model BOVW and sparse coding [8]; and the third is to automatically extract features from images through deep learning methods. Each of the three methods has its own advantages and disadvantages, while the deep learning method does not need to manually extract feature descriptors, and it possesses excellent classification effect, so the trend of using deep learning methods for remote-sensing image scene classification is increasing [9, 10] at present. Among these deep learning methods, traditional convolutional neural network (CNN) is the most widely used one. Compared with traditional handcrafted feature extraction methods, its multistage feature extraction architecture can extract more discriminative semantic features and provides an end-to-end framework. Deep learning techniques for remote-sensing image scene classification are mainly divided into three types, namely unsupervised image classification, supervised image classification, and object-based image analysis [11]. In this paper, the technique of supervised classification is used to classify remote-sensing images.

The article "CAW: A Remote-Sensing Scene Classification Network Aided by Local Window Attention" was published in 2022. Journal: Comput Intell Neurosci.

The difficulty of remote-sensing scene classification is that when determining the scene scheme, (1) the size of key objects varies greatly, (2) many objects unrelated to the scene scheme are often submerged in the image, and (3) compared with natural images, remote-sensing scenes are more complex in terms of spatial arrangement and object distribution [12, 13]. Therefore, how to effectively perceive regions of interest of different sizes and build more discriminative representations from complex object distributions is crucial for understanding remote-sensing scenes.  Figure 1 below shows the changes in the size and number of objects in the aerial images selected in this paper.

In recent years, the transformer has achieved great success in the fields of natural language processing ?NLP?and speech processing (SP). Due to its powerful global feature extraction capability, this structure was introduced into the field of computer vision [14]. The dominant model in the field of computer vision is the CNN network. As the transformer structure becomes more and more efficient, the use of the vision transformer to complete visual tasks has become a new research direction. Vision transformer has powerful global modeling capabilities, but there are some limitations, such as the lack of information exchange in the local area, the large amount of parameters and calculation, getting extremely prone to over-fitting, and the internal structure information of the image block getting destroyed in the process of image patching. In response to the above problems, researchers have redesigned the vision transformer network model. One of the design solutions is to combine the vision transformer and CNN network structure. This network can fuse the global modeling ability of vision transformer and the local feature extraction ability of CNN to improve the model efficiency and performance to a certain extent, such as the conformer [15], CoAtNet [16], visual attention network (VAN [17]), twins [18], and LocalViT [19]. Another method is to control the model capacity by dividing the input feature map into small windows for local-window self-attention. This method can enhance the capture efficiency of local relationships and greatly reduce the computational complexity of the model, such as the Swin transformer [20]. However, it should be noted that in this method, there will be the problem of window limitation. The information of the image only interacts in each small window, and there will be a lack of information interaction between the windows. A Swin transformer uses a shifted window attention to construct the global input image, but it is not constructed in overlapping local windows, so weights can only be shared on channel dimensions and not including global weight sharing on space, and in the form of shifted window attention, it does not really override the relationship between global objects.

The article "CAW: A Remote-Sensing Scene Classification Network Aided by Local Window Attention" was published in 2022. Journal: Comput Intell Neurosci.

For remote-sensing scene classification tasks, it is extremely important to design a network that can learn local and global features to solve the problem of the size change of key targets in each pixel area. The contributions of this paper mainly include the following three points:

1. A parallel model structure is proposed, which spatially solves the problem of limited receptive field of small window self-attention and enhances the spatial-channel modeling capability of the network
2. According to some lightweight vision transformer structures, the computational efficiency has been improved
3. The enhanced classification module is introduced to enhance the feature representation capability of high-level feature remote-sensing image scenes and enhance the expressive capability of the network

Compared with other network structures, this network has higher classification accuracy. Validated on the RSSCN7 dataset and WHU-RS19 dataset, it achieved good results.

The rest of the chapter is structured as follows. The second section is related work, including the research status and analysis of some lightweight convolutional neural network structures and vision transformer structures, as well as the role of parallel structures in feature extraction.  Section 3 provides the method of this paper, including the overall framework of the network and the introduction of each module.  Section 4 shows the experiments of our method on two remote-sensing scene classification datasets. Finally, a conclusion is drawn in Section 5.

The article "CAW: A Remote-Sensing Scene Classification Network Aided by Local Window Attention" was published in 2022. Journal: Comput Intell Neurosci.

## 2. Related Work

### 2.1. Scene Classification Lightweight Network

For the traditional convolutional neural network, the core of the lightweight network is to lighten the network in terms of volume and speed under the premise of maintaining the accuracy as much as possible. For example, the classic convolutional neural network SqueezeNet [21] uses model compression to replace 3 × 3 convolution with 1 × 1 convolution to reduce the amount of parameters and calculation and ShuffleNet [22] proposes pointwise group convolution and channel shuffle to maintain accuracy and reduce the parameters and calculation. MobileNet [23] proposes a depthwise separable convolution structure instead of ordinary convolution, which greatly reduces the model volume and improves the calculation speed. These network structures are widely used in scene classification tasks due to their low computational cost [24].

The introduction of the traditional vision transformer structure into the remote-sensing scene classification task will inevitably introduce a large amount of parameters and calculations. In the existing research, the work of reducing the parameters and calculations of the vision transformer model while maintaining the network accuracy are as follows: The Swin transformer divides the feature map into multiple small windows, adopts the local-window self-attention mechanism in the small windows to reduce the computational complexity, and realizes the global modeling of the image on the channel through the shifted window attention operation and obtains good results; MPViT [25] uses multiscale patch and multipath structure, while reducing the number of channels and reducing model parameters to achieve good performance; CMT [26] introduced depthwise separable convolution in the self-attention module to downsample the feature map, by which computational resources are saved effectively.

This paper refers to the lightweight structure and principles of the convolutional neural network and the vision transformer structure and designs a lightweight network architecture that can combine the advantages of the vision transformer and the convolutional neural network feature extraction.

### 2.2. Transformer Parallel Structure

Parallel structures in neural networks, such as GoogLeNet, [27] improve network performance by paralleling convolution kernels of different sizes (different receptive fields) and Big-Little Net [28] obtains multiscale features by fusing two branches at different scales. According to the structural characteristics of the convolutional network structure and transformer structure, iFormer [29] applies the frequency ramp structure to trade off the high and low frequency components and improves the efficiency through the channel splitting mechanism. In order to be able to learn key objects of different sizes within remote-sensing images and use less amount of parameters and calculation, this paper parallelizes equivalent large convolution kernels with local-window self-attention capturing local relations and global feature extraction.

The article "CAW: A Remote-Sensing Scene Classification Network Aided by Local Window Attention" was published in 2022. Journal: Comput Intell Neurosci.

The channel assignment in the parallel network structure can be divided into two types: one is to compress the channel to a specified number by point convolution, and the other is to divide the channel into a specified number by channel split [30]. Compared with channel split, the method of applying point convolution for channel compression has more parameters. Finally, we split the feature map output by patch merging into two equal parts by channel split and then use channel concatenating and shuffling. The method integrates different features in the branch to realize the construction of global features in the network space-channel range.

## 3. Methodology

### 3.1. Framework Overview

The overall framework of this network structure is shown in Figure 2(a), which consists of three parts: stem, stage, and enhanced classification. Stem consists of convolutional layers and pooling layers, which downscale an input image of size 256 × 256 to 64 × 64. Each stage consists of the patch merging module and CAW module. Patch merging mainly plays the role of downsampling the image, and CAW block is the main feature extraction module. The patch merging module changes the size of the feature map to 1/2 times the original size by selecting elements in the row and column directions of the feature map at intervals of 2 and then stitching them together as a whole tensor. At this time, the channel dimension will become original four times, and a fully connected layer is used to adjust the channel dimension to twice the original to achieve downsampling. After the feature extraction of the three-layer stage, the feature map is input into the enhanced classification layer to obtain the final classification result.

### 3.2. CAW Block

In the task of remote-sensing scene classification, it is of great significance to the classification of remote-sensing scenes to better capture the characteristics of target objects of different sizes and make the features more representative. The concatenation of local-window self-attention mechanism and shifted window self-attention can realize the global modeling of the image in the channel direction. For general image classification tasks, images are generally localized, and this structure can learn most of the content in the image. However, in the scene classification image, there are changes in the size of the target object, so it is particularly important to introduce a global modeling in the space. In the process of using vision transformer to patch the feature map, the internal structure information of the image block will be destroyed, and the feature map is not patched when the convolutional neural network is used to extract the features of the image, which can ensure the integrity of the internal features of the image. Therefore, we consider adding a convolution kernel to the parallel branch for feature extraction. In the convolutional neural network, a larger convolution kernel can achieve more global feature extraction, but a large convolution kernel will bring a huge amount of parameters and calculation, so we introduce the VAN module. The VAN network mainly consists of two parts which are the large kernel attention (LKA) structure and the multilayer perceptron (MLP) structure, where the LKA structure uses a 5 × 5 depthwise convolution, a 7 × 7 depthwise convolution (with a dilation rate of 3), and a 1 × 1 convolution to approximate a 21 × 21 convolution kernel, which can be used in the image with a slight compute costs and parameters to capture long-range relationships.

The article "CAW: A Remote-Sensing Scene Classification Network Aided by Local Window Attention" was published in 2022. Journal: Comput Intell Neurosci.

The CAW block proposed in this paper is a parallel structure module of vision transformer. The Swin transformer divides the feature map into several small windows and then uses the self-attention mechanism for feature extraction for each small window, while the VAN mainly is composed of LKA and MLP. LKA stacks depthwise convolution (DW-Conv), depthwise dilated convolution (DW-D-Conv), and 1 × 1 convolution (1 × 1 Conv) to make LKA equivalent for larger convolutional neural networks. In this paper, a Swin transformer with a window size of 4 × 4 and a VAN network with an equivalent window of 21 × 21 are used to form a parallel structure. This parallel mechanism not only retains the feature extraction advantages of the Swin transformer's local-window self-attention but also makes up the window limit problem for the Swin transformer. The CAW block module diagram is shown in Figure 2(b), and the input feature map channel is divided into two equal parts. The operation description and expressions of the entire network structure are as follows, where X, Y ∈ *R*^*h* × *w* × *c*/2^ are the feature maps obtained by patch merging and channel split.

The feature map of the upper branch converts the feature map of size *H* × *W* × *C*/2 into the feature vector of *HW* × *C*/2 through reshape operation and then uses layer normalization (LN) to normalize the feature vector, and inputs the Swin transformer module for feature extraction; the Swin transformer module is mainly composed of windowed multihead self-attention (W-MSA), moving window multihead self-attention (SW-MSA), MLP, and skip connections. The output formula of the local-window self-attention branch is expressed as

(1) $$\begin{array}{c} X^{\prime }=W-MSA\left(\text{LN}\left(Reshape\left(X\right)\right)\right)+Reshape\left(X\right)\text{,}\\ X_{1}=MLP\left(\text{LN}\left(X^{\prime }\right)\right)+X^{\prime }\text{,}\\ X_{1}^{\prime }=SW-MSA\left(\text{LN}\left(X_{1}\right)\right)+X_{1}\text{,}\\ X_{2}=MLP\left(\text{LN}\left(X_{1}^{\prime }\right)\right)+X_{1}^{\prime }\text{.} \end{array}$$

The feature map of the lower branch enters the VAN for global feature enhancement. In the VAN module, the feature map is first normalized through batch normalization (BN), then through a 1 × 1 convolution kernel,then nonlinearly activated with Gaussian Error Linear Unit (GELU), then through LKA and a 1 × 1 convolution kernel, and finally passes through the MLP structure. The output formula of the global feature supplementary branch is expressed as

(2) $$\begin{array}{c} \begin{array}{c} Y^{\prime }=Conv1\times 1\text{(}LKA\text{(}GELU\text{(}Conv1\times 1\text{(}BN\left(Y\right)\text{)}\text{)}\text{)}\text{)}+Y,\\ Y_{1}=MLP\left(BN\left(Y^{\prime }\right)\right)+Y^{\prime },\\ Y_{1}^{\prime }=Conv1\times 1\text{(}LKA\text{(}GELU\text{(}Conv1\times 1?BN\left(Y_{1}\right)\text{)}\text{)}\text{)}\text{)}+Y_{1,}\\ Y_{2}=MLP\left(BN\left(Y_{1}^{\prime }\right)\right)+Y_{1}^{\prime }. \end{array} \end{array}$$

Finally, merge the feature maps of the two branches and then perform the Shuffle operation to shuffle the feature maps in the two channels so that the feature maps of the two channels are fused. The final output of the module is

(3) $$\begin{array}{c} OUTPUT=Shuffle\left(Concat\left(X_{2},Y_{2}\right)\right)\text{.} \end{array}$$

The article "CAW: A Remote-Sensing Scene Classification Network Aided by Local Window Attention" was published in 2022. Journal: Comput Intell Neurosci.

### 3.3. Enhanced Classification

Current CNNs usually take the final downsampling operation, the fully connected layer, and the softmax classifier as a whole, treating it as a classification layer. Some salient features of this classification layer include those as follows: It usually does not have any convolutional layers, the number of parameters is small, and it is usually a linear feature representation structure. For remote-sensing image scenes, owing to interclass similarity and intraclass variation, it is necessary to highlight local semantics and more discriminative features. Therefore, it is particularly important to optimize the classification layer to have stronger feature representation capabilities. To enhance the feature representation of high-level feature remote-sensing imagery scenes, an additional 1 × 1 convolutional layer and a ReLU activation function are added before the classifier. As shown in Figure 2(c), adding a 1 × 1 convolutional layer before the classifier can increase the nonlinearity of the network and enhance the expressive ability of the network to a certain extent.

## 4. Experiments and Results

### 4.1. Network Complexity

This network is designed based on the vision transformer structure. In order to ensure the accuracy of the network and reduce the amount of parameters and calculation of the network structure, this paper refers to some vision transformer network structures with less parameters and less calculation in the design of the network structure. In order to prove the effectiveness of the network structure proposed in this paper in remote-sensing image classification tasks, this paper selects some classic convolutional neural networks and vision transformer structures for comparative experiments. The comparison table of parameters and calculation is shown in Table 1:

### 4.2. Dataset

This paper conducts experiments on two widely used remote-sensing image classification datasets: RSSCN7 dataset and WHU-RS19 dataset.

The RSSCN7 dataset [34] was released by Qin Zou of Wuhan University in 2015. It contains 2800 remote-sensing images and a total of seven typical scene categories including grassland, forest, farmland, parking, residential, industrial, river, and lake. Each category contains 400 images with a pixel size of 400 × 400, and the diversity of scene images makes it more challenging. In the experiment, we divide the dataset into training sets and test sets in an 8 : 2 ratio by random selection.

The WHU-RS19 dataset [12] was released by Wuhan University in 2011, containing 1005 remote-sensing images and a total of 19 typical scene categories including airports, beaches, bridges, business districts, deserts, farmland, football fields, forests, factories, grassland, mountains, parks, parking, ponds, ports, railway stations, residential, rivers, and viaducts, each of which contains 50 images with a pixel size of 600 × 600. Compared with the RSSCN7 dataset, this dataset is more diverse and has fewer training samples, so it is more challenging. The distribution ratio of training set and test set of this dataset is the same as that of RSSCN7 dataset.

### 4.3. Evaluation Criteria

In this section, we explain the evaluation metrics used to quantify the classification performance of network models: accuracy, precision, sensitivity, specificity, and F1-score. To represent the above metrics, we also need to count four quantities in the confusion matrix: True Positive (TP), True Negative (TN), False Positive (FP), and False Negative (FN). The evaluation index formula is expressed as follows:

(4) $$\begin{array}{c} \begin{array}{c} Accuracy=\frac{TP+TN}{TP+TN+FP+FN},\\ Precision=\frac{TP}{TP+FP},\\ Recall=\frac{TP}{TP+FN},\\ Specificity=\frac{TN}{TN+FP},\\ F1-score=2\times \frac{precision\times recall}{precision+recall} \end{array} \end{array}$$

Confusion matrices are often used to measure model classification performance. This matrix can intuitively reflect the difference between the predicted value and the true value. It consists of four quantities: TP, TN, FP, and FN, which are specifically expressed as follows:

(5) $$\begin{array}{c} \left[\begin{array}{cc} True\;Positive\left(TP\right) & False\;Negative\left(FN\right)\\ False\;Positive\left(FP\right) & True\;Negative\left(TN\right) \end{array}\right]\text{.} \end{array}$$

The article "CAW: A Remote-Sensing Scene Classification Network Aided by Local Window Attention" was published in 2022. Journal: Comput Intell Neurosci.

### 4.4. Preprocessing and Experimental Set-Up

In order to obtain a better training effect, the pictures in the experiment are all subjected to the same preprocessing. First, the pictures in the dataset are scaled and adjusted to 256 × 256, and then the pictures are digitized and normalized. The normalized means set is [0.485, 0.456, 0.406], and standard deviation is set to [0.229, 0.224, 0.225].

The experimental environment of this paper is shown in the following table, including software and hardware information, and the same experimental environment and experimental platform are applied to ensure the fairness and feasibility of the experiment. The training set and test set use the batchsize of 16, and the optimizer uses AdamW, the weight decay coefficient is 5*e* − 2, and the learning rate is 0.0001. The experimental platform data is shown in Table 2.

In the training process, in order to make the network get better convergence effect, a total of 500 epochs were trained in each experiment. We take the highest value of the recognition accuracy of the experimental test set as the final classification accuracy and use the accuracy, sensitivity, precision, specificity, and F1 value as evaluation indicators.

### 4.5. Experimental Results and Discussion

In order to verify that the introduction of VAN based on the structure of Swin transformer can solve the problem of limited receptive field of the Swin transformer and improve the classification effect of remote-sensing scene images, this paper conducts experiments on the RSSCN7 dataset and the WHU-RS19 dataset. Among them, 4 sets of ablation experiments and 10 sets of comparison experiments are set on the RSSCN7 dataset, and 10 sets of comparison experiments are set on the WHU-RS19 dataset. The comparative experiments in this paper include 4 groups of classic convolutional neural networks and 6 groups of transformer structure-related network structures. In order to ensure the accuracy of the experimental results, all experiments in this paper use the same experimental environment, learning rate, loss function, optimizer, batchsize, etc.

The article "CAW: A Remote-Sensing Scene Classification Network Aided by Local Window Attention" was published in 2022. Journal: Comput Intell Neurosci.

In order to study the influence of the depth of CAW on the classification performance of remote-sensing images, we increased the number of module layers at different stages, and compared the accuracy, parameter amount, and computation amount of CAW-Net with different depths, where brackets represent the number of CAW blocks at different stages. The experimental data are shown in Tables 3 and 4:

From the experimental results, with the increase of the number of network layers, the amount of parameters and the amount of calculation increase, the model appears over-fitting, which leads to a decrease in the accuracy rate. Considering both the classification performance and model complexity, we believe that CAW (1, 1, 1) has the best price-performance ratio.

In order to prove the complementarity of the two vision transformer structures and achieve the effect of improving the performance of remote-sensing scene image classification, in the ablation experiment, we split and replace the two branches into four different combined structures to conduct experiments on RSSCN7. The maximum value in the 500 epochs is used as the experimental result, and the experimental results are shown in Table 5. Among them, the Swin transformer-only and VAN-only models are network models obtained by paralleling the same module with other structures unchanged; No Shuffle is the network model obtained by removing the Shuffle structure in the original network structure; and point convolution is a network structure model that replaces the channel segmentation structure in the original network structure with point convolution for channel compression.

It can be seen from Table 5 that the parallel connection of Swin transformer and VAN can solve the problem of limited receptive field of local-windows self-attention and further improve the performance of the network. Compared with using the two modules alone, the accuracy is increased by 0.54% and 1.56%, respectively; Adding Shuffle after the two branches which are connected in parallel can better integrate the features of the two branches, and the network accuracy is increased by 0.89%. In the channel allocation, the spilt operation is better than channel compression, which improves the network performance by 0.72%. Considering the classification performance and model complexity, we believe that this network structure has the best cost performance. In Figure 3, we give the seven-category confusion matrix of the RSSCN7 dataset of this network, and Figure 4 shows the 19-category confusion matrix of this network.

The article "CAW: A Remote-Sensing Scene Classification Network Aided by Local Window Attention" was published in 2022. Journal: Comput Intell Neurosci.

In order to reflect the recognition effect of this network structure on remote-sensing datasets, this paper uses some classic convolutional neural network models and vision transformer network models that perform well in computer vision for comparative experiments. The experiments are performed on the RSSCN7 dataset and the WHU-RS19 dataset under the same environment. The experimental results are shown in Tables 6 and 7. The experimental results with the best effect are marked in bold, and the results are kept to two decimal places.

From the results in Tables 5–7, we can see that compared with other network structures, the network structure proposed in this paper achieves good results on remote-sensing datasets with exponentially reduced parameters and calculation. The parameters of this network are 9.4 times that of ResNet50, 38.8 times that of ViT-Ti, and 12.5 times that of Swin transformer. Compared with these networks, on the RSSCN7 dataset, the accuracy rates of the networks proposed in this paper have increased by 1.79%, 5.36%, and 2.32%, respectively, and the accuracy rates on the WHU-RS19 dataset have increased by 1.46%, 14.08%, and 4.86%.

We apply Gradient-weighted Class Activation Mapping (Grad-CAM) [35] to a different network, using images from the RSSCN7 validation set. Grad-CAM is a recently proposed visualization method, which highlights the feature map in the form of a heat map in order to visualize the feature representation learned by the neural network from an intuitive effect.

As shown in Figure 5, we compare the visualization results of Swin transformer, VAN, and our network. Both the Swin transformer and VAN can capture the area where the target object is located, but it is not accurate enough and there is a certain misjudgment; for example, in the factory scene, the field next to the factory with a similar color is misjudged as a factory. Although VAN can identify the scene area in these scenes, it is more divergent. For example, in the grass and industry scenes, the VAN network can capture the area where the grass and the industry are located, but the range is small and not accurate enough. Our model captures details representing semantic features in complex background images, and it has higher confidence than baseline models in the classification of some difficult objects. We can infer that our model has stronger feature extraction ability and can learn more discriminative features.

The article "CAW: A Remote-Sensing Scene Classification Network Aided by Local Window Attention" was published in 2022. Journal: Comput Intell Neurosci.

## 5. Conclusions

Aiming at the problems of large size changes of key objects, complex spatial arrangement, and object distribution in remote-sensing scene classification tasks, this paper proposes a parallel network model combining the local-window self-attention mechanism and equivalent large convolution kernel. The complementary parallel structure of Swin transformer and VAN realizes the space-channel modeling of transformer network structure with a small amount of parameters and calculation. A series of experiments on two challenging remote-sensing image scene classification datasets show that the network proposed in this paper has good remote-sensing image scene classification results.

In the follow-up work, we will further simplify the network structure and try to optimize the network performance by introducing some other attention mechanismsthat can improve the network performance.

## Figures and Tables

**Figure 1:** (a) and (b) Examples of object size and number variation in remote-sensing images.

**Figure 2:** Network structure diagram.

**Figure 3:** RSSCN7 dataset classification confusion matrix.

**Figure 4:** WHU-RS19 dataset classification confusion matrix.

**Figure 5:** The visualization results (heat maps) of the CAW, Swin transformer, and Van models.

**Table 1:** Comparison of parameters and calculations of the model.

Model	FLOPs (G)	Parameter (M)
ResNet50 [31]	5367.48	23.52
Vgg16 [32]	20185.96	138.36
DenseNet [33]	3742.61	7.98
GoogleNet [27]	2071.13	6.99
ViT-Ti [14]	21980.16	86.38
Swin transformer [20]	7078.50	28.24
VAN [17]	1149.08	41.00
Conformer-Ti [15]	3241.03	11.31
CMT [26]	1580.74	8.17
MPViT [25]	4212.25	6.08
CAW	566.61	1.27

**Table 2:** Experimental platform data.

Attributes	Configuration information
Operating system	Windows 10
CPU	Intel(R) Core (TM) i5-10300H CPU @ 2.50 GHz
GPU	GeForce RTX 2060
CUDA	CUDA 11.6.110
Frame	PyTorch 3.7

**Table 3:** Comparison results of CAW-Net networks with different depths.

Model	Accuracy (%)	Precision (%)	Recall (%)	Specificity (%)	F1-score (%)
CAW (1, 2, 1)	95.18	95.24	95.17	99.21	95.19
CAW (1, 2, 2)	95.54	95.39	95.54	99.29	95.53
CAW (1, 2, 3)	95.35	95.40	95.34	99.24	95.37
CAW (1, 1, 1)	**96.25**	**96.27**	**96.24**	**99.40**	**96.24**

**Table 4:** Comparison of parameters and calculations of CAW-Net with different depths.

Model	FLOPs (G)	Parameter (M)
CAW (1, 2, 1)	656.68	1.58
CAW (1, 2, 2)	695.12	2.03
CAW (1, 2, 3)	733.55	2.48
CAW (1, 1, 1)	566.61	1.27

**Table 5:** Comparison results of parallel networks with different structures.

Model	Accuracy (%)	Precision (%)	Recall (%)	Specificity (%)	F1-score (%)
Swin transformer-only	95.71	95.84	95.73	99.30	95.71
VAN-only	94.69	94.69	94.64	99.14	94.63
No shuffle	95.36	95.39	95.34	99.24	95.36
Point convolution	95.53	95.64	95.53	99.27	95.56
CAW	**96.25**	**96.27**	**96.24**	**99.40**	**96.24**

The article "CAW: A Remote-Sensing Scene Classification Network Aided by Local Window Attention" was published in 2022. Journal: Comput Intell Neurosci.

**Table 6:** Overall accuracy and other parameters of the method on the RSSCN7 dataset.

Model	Accuracy (%)	Precision (%)	Recall (%)	Specificity (%)	F1-score (%)
ResNet50 [31]	94.46	94.59	94.09	99.09	94.49
Vgg16 [32]	93.75	93.79	93.76	98.99	93.71
GoogleNet [27]	93.57	93.61	93.57	98.93	93.56
DenseNet [33]	93.21	93.34	93.21	98.89	93.21
ViT-Ti [14]	90.89	90.89	90.89	98.49	90.89
Swin transformer [20]	93.93	93.96	93.91	99.00	93.93
VAN [17]	94.11	94.17	94.11	99.03	94.11
Conformer-Ti [15]	95.00	95.06	95.00	99.20	95.00
CMT [26]	94.82	95.06	94.83	99.14	94.81
MPViT [25]	95.00	95.03	95.00	99.19	95.00
CAW	**96.25**	**96.27**	**96.24**	**99.40**	**96.24**

**Table 7:** Overall accuracy and other parameters of the method on the WHU-RS19 dataset.

Model	Accuracy (%)	Precision (%)	Recall (%)	Specificity (%)	F1-score (%)
ResNet50 [31]	94.66	95.15	94.62	99.71	94.62
Vgg16 [32]	94.66	95.44	94.61	99.71	94.78
GoogleNet [27]	90.29	90.89	90.50	99.47	90.27
DenseNet [33]	95.15	96.08	95.14	99.73	95.34
ViT-Ti [14]	82.04	83.74	82.11	99.01	82.28
Swin transformer [20]	91.26	92.25	91.35	99.52	91.25
VAN [17]	93.67	94.44	93.72	99.66	93.59
Conformer-Ti [15]	95.63	95.75	95.54	99.76	95.55
CMT [26]	95.63	96.18	95.68	99.76	95.77
MPViT [25]	95.63	95.93	95.75	99.76	95.69
CAW	**96.12**	**96.23**	**96.03**	**99.79**	**95.96**

## Data Availability

The data used to support the findings of this study are available from the corresponding author upon request.
